The article "MicroRNA-19a and microRNA-19b promote the malignancy of clear cell renal cell carcinoma through targeting the tumor suppressor RhoB" was retracted in 2026. Reasons: errors in the data; duplicated data; overlap with earlier publications; original data or images not available.

# MicroRNA-19a and microRNA-19b promote the malignancy of clear cell renal cell carcinoma through targeting the tumor suppressor RhoB

**DOI:** 10.1371/journal.pone.0192790

**Published:** 2018-02-23

**Authors:** Shaoxi Niu, Xin Ma, Yu Zhang, Yen-Nien Liu, Xufeng Chen, Huijie Gong, Yuanxin Yao, Kan Liu, Xu Zhang

**Affiliations:** 1 Department of Urology/State Key Laboratory of Kidney Diseases, Chinese PLA General Hospital/Chinese PLA Medical Academy, Beijing, People's Republic of China; 2 Department of Pathology, Duke University, Durham, North Carolina, United States of America; 3 Graduate Institute of Cancer Biology and Drug Discovery, College of Medical Science and Technology, Taipei Medical University, Taipei, Taiwan; 4 Department of Urology, Dongzhimen Hospital, Beijing University of Chinese Medicine, Beijing, People’s Republic of China; University of South Alabama Mitchell Cancer Institute, UNITED STATES

## Abstract

Clear cell renal cell carcinoma (ccRCC) is the most common subtype of renal cell carcinoma, which shows high aggressiveness and lacks biomarkers. RhoB acts as a tumor suppressor that inhibits the progression of ccRCC. In the present study, we examined the effects of oncogenic microRNAs, miR-19a and miR-19b, on RhoB expression in ccRCC cells. The results showed that both miR-19a and miR-19b could directly target the 3′untranslated region (3’UTR) of RhoB, resulting in the reduced expression of RhoB. With RT-PCR analysis, we detected the increased expression of miR-19a and miR-19b in ccRCC tissues compared to adjacent non-tumor renal tissues. These data also demonstrated an exclusive negative correlation between miR-19a/19b and RhoB expression in ccRCC specimens and cell lines. In addition, the knockdown of RhoB or overexpression of miR-19a and miR-19b in ccRCC cells could promote cell proliferation, migration and invasion. These data demonstrate the direct roles of miR-19a and miR-19b on the repression of RhoB and its consequences on tumorigenesis, cancer cell proliferation and invasiveness. These results suggest the potential clinical impact of miR-19a and miR-19b as molecular targets for ccRCC.

## Introduction

Renal cell carcinoma (RCC) is the second leading cause of cancer death in patients with urological tumors, and accounts for approximately 3% of adult malignancies [1]. The overall incidence and mortality of RCC have significantly increased over the past 20 years. Among all RCC cases, approximately 70%~ 80% subtypes are clear cell renal cell carcinoma (ccRCC). Surgery is the primary treatment for patients with localized ccRCC [2]. For patients with relapsed or metastasized tumors, clinical treatment options are extremely limited because ccRCC is often resistant to chemotherapy and radiotherapy [3]. In addition, there are no diagnostic and therapeutic biomarkers currently available for this disease, and ccRCC patients are often diagnosed at late stages with poor prognosis for clinical outcomes [4]. Thus, there is a clear need to identify biomarkers for early diagnosis and molecular targets for establishing novel therapeutic strategies for ccRCC.

The article "MicroRNA-19a and microRNA-19b promote the malignancy of clear cell renal cell carcinoma through targeting the tumor suppressor RhoB" was retracted in 2026. Reasons: errors in the data; duplicated data; overlap with earlier publications; original data or images not available.

The Rho protein family is a subgroup of small GTPases of the Ras superfamily, comprising twenty members. Rho family proteins regulate a variety of cell functions, including actin organization and cell shape, cell adhesion, cell motility, membrane trafficking and gene expression [5]. A recent study has also indicated that Rho family proteins play an important role in angiogenesis [6]. Interestingly, while other Rho proteins function as oncogenic proteins, RhoB acts as a tumor suppressor in cancer cells [7]. Studies have shown that the decreased expression of RhoB protein in solid tumors correlates with tumor staging [8], and the overexpression of RhoB increases apoptosis and decreases the migration, invasion and metastasis of cancer cells [9, 10]. In addition, recent studies have shown that targeting RhoB could inhibit the tumor growth of colorectal cancer and hepatocellular carcinoma in mouse xenograft models [11, 12, 13]. Consistent with these observations, in a previous study, we demonstrated that ccRCC tumors have lower RhoB protein levels, and the overexpression of RhoB can inhibit cancer cell proliferation and survival [14]. These results thus indicate the potential of RhoB as a therapeutic target for cancer treatment.

MiRNAs play vital roles in tumor progression and metastasis in many tumors, including kidney cancer [2, 3, 15, 16]. MicroRNAs bind to the 3’-untranslated region (3’-UTR) of target mRNAs and thus function as regulators for gene expression at the post-transcriptional level [17]. In colorectal cancer and hepatocellular carcinoma cells, studies have showed that miR-21 can regulate RhoB protein expression [11, 12]. To explore whether other miRNAs also target and regulate the protein expression of RhoB mRNA, we used miRNA target prediction algorithms with miRDB, TargetScan and PicTar to search for RhoB-targeting miRNAs. The results showed that miR-21 is listed in the top miRNA candidates that may have potential for RhoB-targeting. Moreover, we observed that miR-19a and miR-19b have the highest scores for RhoB-targeting potential in this bioinformatics analysis. MiR-19a and miR-19b belong to the miR-17–92 cluster located on chromosome 13q31.3 and have been implicated as tumor-associated miRNAs involved in tumorigenesis[18]. The miR-17–92 cluster has also been implicated in initiating carcinogenesis in B cell lymphoma and targeting proapoptotic genes, such as PTEN, E2F1, and Bcl2l11/BIM [19, 20]. Previous studies have shown that miR-19a and miR-19b are involved in the carcinogenesis and cancer development of different human cancers, including B-cell lymphomas [21], breast cancer [22] and cervical cancer [23]. Other studies have also demonstrated that miR-19a and miR-19b directly target SOCS-1 (suppressor of cytokine signaling 1), a gene that shows loss of function in multiple myeloma, and inhibits IL-6 growth signaling[24]. However, whether miR-19a and miR-19b target and regulate the expression of RhoB in ccRCC remains unknown.

The article "MicroRNA-19a and microRNA-19b promote the malignancy of clear cell renal cell carcinoma through targeting the tumor suppressor RhoB" was retracted in 2026. Reasons: errors in the data; duplicated data; overlap with earlier publications; original data or images not available.

In the present study, we examined the potential regulatory effects of miR-19a and miR-19b on RhoB protein expression and characterized their biological roles in ccRCC cells. We examined the levels of RhoB mRNA, miR-19a and miR-19b in ccRCC in paired tumor and non-tumor specimens and ccRCC cell lines. These data demonstrated that miR-19a and miR-19b can directly inhibit RhoB expression, resulting in consequent biological effects on the tumorigenesis, proliferation, and invasiveness of ccRCC cells.

## Materials and methods

### Ethics statement

The protocol for the present study was approved by the Protection of Human Subjects Committee, Chinese People’s Liberation Army (PLA) General Hospital. All patients enrolled in the present study provided signed informed consent. Specimens from human subjects were collected from May to December 2013, and the experiments conducted with these human specimens were initiated on January 2014.

### Patients and samples

Seventy patients diagnosed with clear cell renal cell carcinoma and treated with surgery in the Department of Urology of the Chinese PLA General Hospital in 2013 were enrolled in the present study. Paired tumor tissues and adjacent non-tumor kidney tissues were collected and added to the kidney cancer tissues bank after clinical and pathological confirmations. All tissue samples were preserved with flash freezing in liquid nitrogen after resection and stored at −80 °C. Patients who received radical nephrectomy in our hospital, with pathologic diagnosis of ccRCC, and both tumor and normal renal tissues available after surgery were included in the present study. Patients receiving chemotherapy or radiotherapy prior to surgery, or patients with multiple renal tumors or distant metastasis were excluded. TNM staging of ccRCC samples was assessed according to the 7th edition of the AJCC Cancer Staging Manual [25], and the Fuhrman nuclear grading system was used to determined nuclear grades. The clinical characteristics of the enrolled patients are shown in Table 1. All authors had access to information on the identities of individual participants during data collection.

The article "MicroRNA-19a and microRNA-19b promote the malignancy of clear cell renal cell carcinoma through targeting the tumor suppressor RhoB" was retracted in 2026. Reasons: errors in the data; duplicated data; overlap with earlier publications; original data or images not available.

**Table 1:** The correlation between miR-19a and miR-19b expression and clinical and pathological parameters of ccRCC patients.

Variables	Total(n = 67)	miRNA expression		P-value
		miR-19a	miR-19b	
Age(years)				
<55	35	0.032±0.009	0.030±0.008	0.3667 (miR-19a)
≥55	32	0.044±0.001	0.040±0.010	0.1507 (miR-19b)
Tumor volume				
≤ 150(cm^3^)	42	0.011±00.03	0.011±0.003	<0.01 (miR-19a)
>150(cm^3^)	25	0.083±0.013	0.084±0.013	<0.01 (miR-19b)
TNM stage				
1	52	0.026±0.006	0.020±0.006	<0.01 (miR-19a)
2–4	15	0.092±0.017	0.093±0.016	<0.01 (miR-19b)
Fuhrman stage				
G1-2	49	0.022±0.006	0.022±0.007	<0.01 (miR-19a)
G3-4	18	0.082±0.015	0.083±0.014	<0.01 (miR-19b)

### Cell culture and reagents

Human renal cancer cell lines 786-O, Caki-1, Caki-2, A498, SN12pm6, and ACHN, and normal renal cell lines HKC and HK2 were purchased from the National Platform of Experimental Cell Resources for Sci-Tech (Beijing, China). The cells were cultured in RPMI 1640/DMEM/MEM medium (Thermo Fisher, NY, CA)supplemented with 10% fetal bovine serum (Invitrogen, Carlsbad, CA), 100 U/ml of penicillin and 100 U/ml of streptomycin (Invitrogen, Carlsbad, CA). All cell lines were maintained in a sterile incubator with a mixture of 95% air and 5% CO2 at 37°C.

### RNA isolation and quantitative real-time PCR

Total RNA was extracted from tissues or cells using Trizol reagent (Invitrogen, Carlsbad, CA) according to the manufacturer’s instructions. The TransScript Kit (TransGen Biotech Co., Beijing, China) was used for RT-PCR for RhoB. M-MLV (TIANGEN Biotech Co, Beijing, China) was used to synthesize the complementary DNA templates for miRNA. The quantification of both RhoB gene and miRNA expression was performed on an ABI PRISM 7500 Sequence Detection System (Applied Bio systems, Foster City, CA) with SYBR Green (TransGen Biotech Co., Ltd, Beijing, China). The relative expression of both mRNA and miRNA was determined by using the ΔΔCt method. The expression of RhoB was normalized to the expression of human peptidylprolyl isomerase A (PPIA), and the level of miRNA was normalized to U6. The primers used in real-time RT-PCR are shown in Table 2.

**Table 2:** Primer sequences used in the present study.

Primer name	
Universe Reverse	CTCACAGTACGTTGGTATCCTTGTG
miR-19a RT	CTCACAGTACGTTGGTATCCTTGTGATGTTTCGATGCCATATTGTACTGTGAGTCAGTTTT
miR-19a Forward	ACACTCCAGCTGGGTGTGCAAATCCATGCAA
miR-19b RT	CTCACAGTACGTTGGTATCCTTGTGATGTTTCGATGCCATATTGTACTGTGAGTCAGTTTT
miR-19b Forward	ACACTCCAGCTGGGTGTGCAAATCCATGCAA
RhoB Forward	GCCTGTCCTAGAAGTGAA
RhoB reverse	GAATGCTACTGTCGTATGC

The article "MicroRNA-19a and microRNA-19b promote the malignancy of clear cell renal cell carcinoma through targeting the tumor suppressor RhoB" was retracted in 2026. Reasons: errors in the data; duplicated data; overlap with earlier publications; original data or images not available.

### Antibodies and western blotting

The anti-RhoB antibody was obtained from Proteintech (Chicago, USA), anti-cleaved caspase-9 antibody was purchased from Epitomics (Burlingame, CA), and anti-β-actin antibody was obtained from ZSGB-BIO (Beijing, China). Preparation of the total cell lysate and Western blot analysis were conducted with standard techniques as previously described [14].

### Transfection and luciferase assay

The full-length RhoB 3’-UTR-luciferase reporter and its negative control vector psi-check2 were provided by Dr. Rossi (Department of Molecular Biology, Beckman Research Institute of the City of Hope). The has-miR-19a and has-miR-19b mimics, control oligo (NC), has-miR-19a and has-miR-19b inhibitors, miRNA inhibitor control, and small interfering RNA (siRNA) targeting RhoB (RhoB siRNA: Sense: 5’-ACGUCAUUCUCAUGUGCUUTT-3’; Anti-sense: 5’-AAGCACAUGAGAAUGACGUTT) were all chemically synthesized by Shanghai Gene-Pharma Co. (Shanghai, China). For the mutagenesis of miRNA target sites in the 3’-UTR region of the reporter, mutations were introduced into the seed sequence by using the QuikChange Site-Directed Mutagenesis Kit II (Stratagene, USA) according to the manufacturer’s protocol. Mutations were confirmed by sequencing at Genewiz (Suzhou, China). The RNA oligonucleotides transfections were performed with Lipofectamine 2000 (Invitrogen, Carlsbad, CA) according to the manufacturer’s protocol. For Luciferase Assay, A498 or 786-O cells were plated in 24-well plates. After 24 hours, the cells were cotransfected with oligos of miRNA mimics (0.6 ug), miRNA inhibitor (0.6 ug) or negative control (0.6 μ g) together with the appropriate reporter plasmid (0.2 ug). After 48 hours, the Dual-Glo Luciferase Assay System (Promega, Madison USA) was used to measure the luciferase activity on a Centro XS3 LB960 luminometer (Berthold, USA), according to the manufacturer’s instructions. The ratio of Rluc/Fluc was used to measure the repression efficiency.

### Wound healing assay and plate colony formation assay

For wound healing assays, the cells were seeded onto six-well plates at 24 hours post-transfection. Confluent monolayer cells were scratched by a 200-ul pipette tip, and then washed three times with PBS. After fresh serum-free medium was replaced, wound closure was photographed at 0, 12, and 24 hours at the same position. For the colony formation assay, cells transfected with plasmid and mimics were seeded onto six-well plates (300 cells per well) and cultured at 37°C for 14 days. The cells were fixed with 70% methanol for 15 minutes and subsequently stained with 0.2% crystal violet. The number of positive colonies (consisting of more than 50 cells) was counted after 4 weeks of growth.

The article "MicroRNA-19a and microRNA-19b promote the malignancy of clear cell renal cell carcinoma through targeting the tumor suppressor RhoB" was retracted in 2026. Reasons: errors in the data; duplicated data; overlap with earlier publications; original data or images not available.

### Cell proliferation and migration analyses

Cell proliferation was measured by MTS assay using an ELx800 plate reader (BioTek, USA) with the CellTiter 96 Aqueous One Solution (Promega, Madison, USA). Cell migration assay was conducted with an 8 mm–pore size membrane Transwell apparatus (Corning Costar Corp, Cambridge, USA). These assays were performed as previously described [14].

### Flow cytometry analysis

Cell apoptosis were measured by flow cytometry analysis. Briefly, 1x10^6^ cells were stained with Annexin V-PE (Annexin V-PE kit, BD Biosciences, USA), and apoptotic cells were counted on a FACSCalibur Flow Cytometer (BD Biosciences, USA). The data were analyzed using CellQuest Pro software (BD Biosciences, USA). Up to 5x10^5^ cells were analyzed for each sample.

### Statistical analysis

All statistical analyses were performed with SPSS statistical software 13.0 (SPSS Inc., Chicago, IL), and the statistical significance was set at P<0.05. ANOVA and Student’s t-test were used as appropriate for all results.

## Results

### Negative collection between miR-19a/19b and RhoB in ccRCC specimens and cell lines

To validate whether miR-19a and miR-19b functionally regulate the expression of RhoB, we examined the expression of miR-19a, miR-19b and RhoB in patient tumor tissue samples (Fig 1A). The results showed that compared to the non-cancerous tissues ccRCC tumor tissues have a higher level of miR-19a and miR-19b (p<0.05). Moreover, relatively lower amounts of RhoB mRNA were detected in these tumor tissues. Notably, some tumor tissues had low endogenous miR-19a and miR-19b expression when compared to paired non-tumorous tissues (Fig 1B), and these tumor tissues expressed relatively high levels of RhoB protein (Fig 1C). The relative expression of miR-19a,miR-19b and RhoB in paried specimens individually showed in the supplementary information.(S1 Fig).The mRNA levels of miR-19a and miR-19b in ccRCC cell lines were also dramatically inversely correlated to RhoB expression among normal renal cells (HK2 and HKC) and ccRCC cell lines (A498, Caki-2, 786-O, ACHN, Caki-1, and SN12) (Fig 1D). Moreover, the protein levels of RhoB were increased in normal renal cells compared to those in ccRCC cell lines (Fig 1E). These results provide strong evidence to support the hypothesis that RhoB is a tumor suppressor in ccRCC, and miR-19a and miR-19b may act as oncomirs and down-regulate RhoB expression in ccRCC through a post-transcriptional mechanism.

**Fig 1:** miR-19a/19b and RhoB expression levels are negatively correlated in patient tissues samples and cell lines. (A) QRT-PCR analysis for miR19a/b and RhoB expression in paired patient specimens (n = 70). (B) QRT-PCR analysis for miR19a/b in patient specimens (n = 8). (C) Western blot analysis for RhoB expression in the same specimens as panel B. N1-8 are normal tissues and A1-8 are paired tumor tissues. (D and E) QRT-PCR and Western blot analysis for miR19a/b and RhoB expression in normal renal cells and ccRCC cell lines. β-actin was used as loading control for western blot. The data represent the average of three independent experiments. *Indicates statistical significance (P<0.05).

The article "MicroRNA-19a and microRNA-19b promote the malignancy of clear cell renal cell carcinoma through targeting the tumor suppressor RhoB" was retracted in 2026. Reasons: errors in the data; duplicated data; overlap with earlier publications; original data or images not available.

### Correlations of miR-19a and miR-19b with clinical features

We next analyzed the correlations of miR-19a and miR-19b expression and the clinical features of ccRCC. A total of 47 males and 20 females were included in this analysis. The data showed that the expression of the these two miRNAs was significantly positively associated with tumor size (P<0.001), TNM stage (P<0.001) and Fuhrman tumor grade (P<0.001, Table 1). However, no significant correlation was observed between miRNA expression and patients’ age (p = 0.3667).

### MiR-19a and miR-19b inhibit RhoB at both the mRNA and protein levels

To further confirm the relationship between miR-19a and miR-19b and RhoB, we examined the expression of RhoB in cells after transfection with miR-19a and miR-19b mimics. QRT-PCR and western blot analysis further supported the down-regulatory effect of miR-19a and miR-19b on the protein levels of RhoB in ccRCC cells (Fig 2A). In contrast, cells transfected with hsa-miR-19a and miR-19b inhibitors showed the increased expression of RhoB (Fig 2B). The bioinformatics analyses showed a potential binding ability for both miR-19a and miR-19b to the 3’-UTR region of RhoB (857–864 base pairs (bp), Fig 2C). Interestingly, the miR-19a and miR-19b binding site in RhoB is a highly conserved sequence motif located between 857 and 864 bp of the RhoB 3’UTR. Based on these findings, we performed a luciferase reporter assay to examine the regulatory effects of miR-19a and miR-19b on the gene post-transcription of RhoB. We co-transfected RhoB 3’-UTR-luciferase reporter and miR-19a and miR-19b mimics into A498 cells. The transfection of miR-19a and miR-19b mimics dramatically decreased the relative luciferase activity of the reporter containing the wild-type RhoB 3’-UTR region (RhoB-3’UTR-wt). However, the co-transfection of miR-19a and miR-19b mimics did not show obvious effects on the luciferase activity of the reporter when the RhoB 3’-UTR region was mutated (RhoB-3’UTR-mut) (Fig 2D). In addition, has-miR-19a and miR-19b inhibitors and RhoB-3’UTR-wt or RhoB-3’UTR-mut were co-transfected into 786-O cells, and the luciferase activity was determined. We found that the co-transfection of has-miR-19a and miR-19b inhibitors increased the luciferase activity of RhoB-3’UTR-wt but had no effect on the luciferase activity of RhoB-3’UTR-mut (Fig 2E). These data suggest that miR-19a and miR-19b suppress RhoB expression by direct binding to the 3’UTR of RhoB.

The article "MicroRNA-19a and microRNA-19b promote the malignancy of clear cell renal cell carcinoma through targeting the tumor suppressor RhoB" was retracted in 2026. Reasons: errors in the data; duplicated data; overlap with earlier publications; original data or images not available.

**Fig 2:** miR-19a and miR-19b regulate RhoB expression. (A and B) QRT-PCR analysis for miR19a/b (top) and Western -blot analysis of RhoB (bottom) expression in A498 and 786-O cells after transfection with miR-19a and miR-19b mimics or inhibitors for 48 h. Control mimics or inhibitors were included as a negative control. β-actin was included for equal protein loading. (C) The predicted binding motif sequence of miR-19a and miR-19b in the 3’-UTR region of RhoB. (D) Reporter assay showing the effect of miR19a/b mimics on the luciferase activity of reporter plasmids containing RhoB-3’UTR-wt, RhoB-3’UTR-mut or empty plasmid psi-check2 in A498 cells transfected with miR19a/b mimics. Control oligo was included as a negative control. (E) Reporter assay showing the effect of miR-19a and miR-19b inhibitors on luciferase activity of reporter plasmids containing RhoB-3’UTR-wt, RhoB-3’UTR-mut or empty plasmid psi-check2 in 786-O cells. The data represent the average of three independent experiments. *Indicates statistical significance (P<0.05).

### MiR-19a and miR-19b overexpression and RhoB knockdown show similar phenotypes in promoting cell growth, invasion, and migration

We further tested whether the interaction of miR-19a and miR-19b with RhoB plays a role in the proliferation and progression of ccRCC cells. We performed MTS assay to evaluate the potential growth promoting effects of miR-19a and miR-19b on the cell growth of ccRCC. The efficiency of RhoB knockdown was showed in S2 Fig. The results showed that the overexpression of miR-19a and miR-19b mimics remarkably enhanced the proliferation potential of A498 cells (Fig 3A). The expression of RhoB was lower with the transfection of si-RhoB both at mRNA and protein level (S2 Fig). The clonogenic survival assay also showed that the overexpression of miR-19a and miR-19b mimics increased the colony formation of A498 cells (Fig 3B). In addition, the transfection of miR-19a and miR-19b mimics in A498 cells enhanced the migration and invasiveness of A498 cells (Fig 3C and 3D). These similar results were observed in cells with RhoB knockdown by RhoB-siRNA transfection (Fig 3E). These data suggest that miR-19a and miR-19b promote ccRCC cell proliferation, motility, and migration through direct targeting of the RhoB tumor suppressor.

**Fig 3:** Overexpression of miR-19a and miR-19b or RhoB knockdown show similar phenotypes in promoting the growth, migration and mobility of ccRCC cells. (A) MTS results showing the promotion potential of miR-19a and miR-19b mimics overexpression or RhoB knockdown on the proliferation of A498 cells. (B) Representative images and quantification show the clonogenic plating efficacy of A498 cells overexpressing miR-19a and miR-19b mimics. (C and D) Representative images (right) and quantification (left) of wound healing assay (C) and transwell assay (D) showing the potential effects of the overexpression of miR-19a and miR-19b mimics on the migration and invasiveness of the cells. Control oligo was included as a negative control. (E and F) Representative images (right) and quantification (left) of wound healing assay (E) and transwell assay (F) showing the potential effects of RhoB knockdown on the migration and invasiveness of the cells. Control siRNA was included as a negative control. The data are representative of three independent experiments performed in triplicate. *Significant differences from control oligo-transfected cells (P<0.05).

The article "MicroRNA-19a and microRNA-19b promote the malignancy of clear cell renal cell carcinoma through targeting the tumor suppressor RhoB" was retracted in 2026. Reasons: errors in the data; duplicated data; overlap with earlier publications; original data or images not available.

### MiR-19a and miR-19b inhibitors induce cell growth, migration, and invasiveness of 786-O cells

To investigate whether the miR-19a and miR-19b inhibitors could have potential inhibitory effects on the migration and invasiveness of ccRCC cells, we transfected 786-O cells with miR-19a and miR-19b inhibitors or inhibitor control oligo. Interestingly, transfection with miR-19a and miR-19b inhibitors resulted in the dramatically decreased migration and reduced invasiveness of 786-O cells (Fig 4A and 4B). To determine the effects of miR-19a and miR-19b inhibitors on cell proliferation features, we performed MTS assay of 786-O cells transfected with miR-19a and miR-19b inhibitors or inhibitor control oligo. The results showed that transfection with miR-19a and miR-19b inhibitors led to significantly reduced cell growth (Fig 4C). These data are similar to those of a previous study showing the overexpression of RhoB in 786-O cells [14], which further supports the hypothesis that miR-19-RhoB signaling axis regulates the migration, invasiveness, and proliferation of ccRCC cells.

**Fig 4:** MiR-19a and miR-19b inhibitors reduce cell migration and invasiveness, and inhibit cell proliferation. (A) Representative images showing that the transfection of miR-19a and miR-19b inhibitors decreases the migration of 786-O cells by wound healing assay (Left); quantification of relative migration at 12 and 24 h (Right). (B) Representative images and quantification of relative migration, showing that the transfection of miR-19a and miR-19b inhibitors reduces the invasiveness of 786-O cells by transwell assay. The migratory activities of 786-O cells transfected with control oligo were was included as a negative inhibitor control. (C) The proliferation potential of 786-O cells transfected with miR-19a and miR-19b inhibitors or control oligo was determined by the MTS Assay. The data are representative of three independent experiments. *Significant differences from control oligo-transfected cells (P<0.05).

The article "MicroRNA-19a and microRNA-19b promote the malignancy of clear cell renal cell carcinoma through targeting the tumor suppressor RhoB" was retracted in 2026. Reasons: errors in the data; duplicated data; overlap with earlier publications; original data or images not available.

### Effect of miR-19a and miR-19b on cell apoptosis

We further determined the effect of miR-19a and miR-19b on apoptosis in ccRCC cells. Apoptosis is a crucial event during malignant transformation [26], and we previously showed that RhoB overexpression could influence the apoptosis of ccRCC cells [14]. In the present study, we treated 786-O cells with miR-19a and miR-19b inhibitors and showed that transfection with miR-19a and miR-19b inhibitors resulted in significant increases of apoptosis as determined by Annexin V-PE staining (Fig 5A). We also examined changes in caspase-9, an apoptotic protein in these cells, and found that the cleavage of caspase-9 was increased in 786-O cells transfected with miR-19a and miR-19b inhibitors (Fig 5B). These results demonstrated that levels of miR-19a and miR-19b affect the apoptosis of ccRCC cells.

**Fig 5:** MiR-19a and miR-19b inhibitors induce cell apoptosis. (A) Flow cytometry results of Annexin-V5 analysis in 786-O cells transfected with miR-19a and miR-19b inhibitors. An inhibitor control was included as a negative control. Graphs showing changes of the apoptotic percentage of the cells (left); quantification of relative apoptosis (right). The data represent the means ± S.D. from three independent experiments performed in triplicate. *Significant differences from control oligo-transfected cells (P<0.05) (B) Western blot results showing the effect of miR-19a and miR-19b inhibitors on the expression of cleaved caspase-9 in 786-O cells. (C) Potential mechanism showing the effect of the negative regulation of RhoB by miR-19a/b on the proliferation, migration, invasion and apoptosis of ccRCC.

## Discussion

In the present study, we investigated the potential regulatory effects of miR-19a and miR-19b on RhoB expression and examined its consequences on the biological behavior of ccRCC cells (Fig 5C). We observed the increased expression of miR-19a and miR-19b in tumor tissues compared to that in paired and adjacent normal tissues, and this expression was inversely correlation with RhoB expression. We also identified a similar inverse correlation between miR-19a and miR-19b and RhoB expression in established ccRCC cell lines. In addition, the overexpression or inhibition of miR-19a and miR-19b respectively led to a decrease or increase of RhoB. Luciferase reporter assay further showed that the transfection of miR-19a and miR-19b inhibitors into ccRCC cells significantly suppressed RhoB 3’-UTR luciferase-reporter activity. Thus, these results suggest that miR-19a and miR-19b can directly and inversely regulate RhoB gene expression. Interestingly, these data further showed that transfection with miR-19a and miR-19b mimics or RhoB-siRNA increased the viability and migration of A498 cells, and transfection with miR-19a and miR-19b inhibitors showed inverse effects in 786-O cell lines. Moreover, the down–regulation of miR-19a and miR-19b remarkably induces the apoptosis of ccRCC cells and increases the levels of cleaved apoptotic casp9 protein. These data suggest the potential effects of miR-19a and miR-19b on cancer cell invasiveness and metastasis via targeting the RhoB tumor suppressor.

The article "MicroRNA-19a and microRNA-19b promote the malignancy of clear cell renal cell carcinoma through targeting the tumor suppressor RhoB" was retracted in 2026. Reasons: errors in the data; duplicated data; overlap with earlier publications; original data or images not available.

Rho GTPases have been implicated in tumor development and progression. Previous studies have shown that the levels of both Rho GTPase mRNA and protein expression were correlated with tumor progression [27]. Rho GTPase family proteins, such as Ras, Rac1 and Cdc42, enhance oncogenesis, invasion and metastasis [28]. However, recent studies have indicated that RhoB, unlike its other family proteins, RhoA and RhoC, whose expression is up-regulated in different types of human cancers, may play a role as a tumor suppressor [13, 29]. One potential mechanism is that RhoB competes for binding to Rho effector proteins and interferes with oncogenic signaling by Rho [30]. Other studies have shown that RhoB expression changes the apoptotic response of transformed cells to FTI (Farnesyltransferase inhibitor), DNA damaging agents and paclitaxel [10,13]. Thus, RhoB could act as a death effector or modifier in downstream or paralleled signaling to the DNA-damage-response pathway.

MiRNAs can act as “oncomirs” or “tumor suppressors” in cancer progression [3]. Studies have shown that miRNAs, such as miR-203a, miR-21, miR-17, miR-23 and miR-199a, are also involved in the progression of ccRCC [3]. A previous study reported that the oncogenic miR-17-92 cluster is frequently up-regulated in human cancers and plays a role in tumorigenesis [31, 32]. MiR-19a and miR-19b are two important miRNAs in this cluster, and these molecules could regulate the expression of tumor suppressor genes in lymphoma cells [20]. Both miR-19a and miR-19b were also highly expressed in gliomas [18] and could regulate the cell proliferation and invasion of cervical carcinoma through targeting CUL5 [23]. Notably, RhoB activity has been identified by biochemical studies, suggesting that the GTP-binding/GTP-hydrolysis cycle is tightly regulated by RhoB and is essential for the regulation of Rho family GTPase activities. Studies have further shown that the activities of classic regulators, such as guanine nucleotide exchange factors, GTPase-activating proteins, and Rho GTPase, can be controlled by miRNAs, such as miR-21[11].

The article "MicroRNA-19a and microRNA-19b promote the malignancy of clear cell renal cell carcinoma through targeting the tumor suppressor RhoB" was retracted in 2026. Reasons: errors in the data; duplicated data; overlap with earlier publications; original data or images not available.

In conclusion, the present study provides evidence for novel regulators, miR-19a and miR-19b, of RhoB expression, which plays important roles in the development of malignant ccRCC via promoting cell proliferation, migration and invasiveness. These data also show the impact of miR-19a and miR-19b as potential diagnostic biomarkers and therapeutic targets on clinical management for ccRCC.

## Supporting information

S1 Fig The individual expression of the miR-19a, miR-19b and RhoB in specimens. (TIF)

S2 Fig The efficiency of RhoB knockdown. (TIF)

## References

[1] MaX, FanY, GaoY, ZhangY, HuangQ, AiQ, et al, Dicer is down-regulated in clear cell renal cell carcinoma and in vitro Dicer knockdown enhances malignant phenotype transformation, Urol Oncol, 32 (2014) 46 e49–17.10.1016/j.urolonc.2013.06.01124094887

[2] WhiteNM, KhellaHW, GrigullJ, AdzovicS, YoussefYM, HoneyRJ, et al, miRNA profiling in metastatic renal cell carcinoma reveals a tumour-suppressor effect for miR-215, Br J Cancer, 105 (2011) 1741–1749. doi: 10.1038/bjc.2011.401 2203327210.1038/bjc.2011.401PMC3242591

[3] Al-AliBM, RessAL, GergerA, PichlerM, MicroRNAs in renal cell carcinoma: implications for pathogenesis, diagnosis, prognosis and therapy, Anticancer Res, 32 (2012) 3727–3732. 22993312

[4] HuangQB, MaX, ZhangX, LiuSW, AiQ, ShiTP, et al, Down-Regulated miR-30a in Clear Cell Renal Cell Carcinoma Correlated with Tumor Hematogenous Metastasis by Targeting Angiogenesis-Specific DLL4, PLoS One, 8 (2013) e67294 doi: 10.1371/journal.pone.0067294 2382625810.1371/journal.pone.0067294PMC3694928

[5] HeasmanSJ, RidleyAJ. Mammalian Rho GTPases: new insights into their functions from in vivo studies. Nat Rev Mol Cell Biol. 2008;9:690–701. doi: 10.1038/nrm2476 1871970810.1038/nrm2476

[6] ChenW, MaoK, LiuZ, Dinh-XuanAT, The role of the RhoA/Rho kinase pathway in angiogenesis and its potential value in prostate cancer.Oncol Lett. 201410.3892/ol.2014.2471PMC418656025289078

[7] PrendergastGC, Actin’ up: RhoB in cancer and apoptosis, Cancer,11 (2001)162–168.10.1038/3510109611905808

[8] RidleyAJ, Rho proteins and cancer, 84 (2004)13–19.10.1023/B:BREA.0000018423.47497.c614999150

[9] JiangK, SunJ, ChengJ, DjeuYJ, WeiS, SebtiS, Akt mediates Ras downregulation of RhoB, a suppressor of transformation, invasion, and metastasis, Mol Cell Biol, 24 (2004) 5565–5576. doi: 10.1128/MCB.24.12.5565-5576.2004 1516991510.1128/MCB.24.12.5565-5576.2004PMC419878

The article "MicroRNA-19a and microRNA-19b promote the malignancy of clear cell renal cell carcinoma through targeting the tumor suppressor RhoB" was retracted in 2026. Reasons: errors in the data; duplicated data; overlap with earlier publications; original data or images not available.

[10] AxLiu, DuW, LiuJP, JessellTM, PrendergastGC. RhoB alteration is necessary for apoptotic and antineoplastic responses to farnesyltransse inhibitors,Mol Cell Biol,16(2000)6105–611310.1128/mcb.20.16.6105-6113.2000PMC8608610913192

[11] LiuM, TangQ, QiuM, LangN, LiM, ZhengY, et al, miR-21 targets the tumor suppressor RhoB and regulates proliferation, invasion and apoptosis in colorectal cancer cells, FEBS Lett, 585 (2011) 2998–3005. doi: 10.1016/j.febslet.2011.08.014 2187259110.1016/j.febslet.2011.08.014

[12] ConnollyEC, Van DoorslaerK, RoglerLE, RoglerCE, Overexpression of miR-21 promotes an in vitro metastatic phenotype by targeting the tumor suppressor RHOB, Mol Cancer Res, 8 (2010) 691–700. doi: 10.1158/1541-7786.MCR-09-0465 2046040310.1158/1541-7786.MCR-09-0465

[13] LiuAX, RaneN, LiuJP, PrendergastGC, RhoB is dispensable for mouse development, but it modifies susceptibility to tumor formation as well as cell adhesion and growth factor signaling in transformed cells, Mol Cell Biol, 21 (2001) 6906–6912. doi: 10.1128/MCB.21.20.6906-6912.2001 1156487410.1128/MCB.21.20.6906-6912.2001PMC99867

[14] ChenWH, NiuSX, MaX, ZhangP, GaoY, FanY et al, RhoB Acts as a Tumor Suppressor That Inhibits Malignancy of Clear Cell Renal Cell Carcinoma, PLoS One, 11 (2016) e0157599 doi: 10.1371/journal.pone.0157599 2738422210.1371/journal.pone.0157599PMC4934884

[15] OuyangM, LiY, YeS, MaJ, LuL, LvW, et al, MicroRNA profiling implies new markers of chemoresistance of triple-negative breast cancer, PLoS One, 9 (2014) e96228 doi: 10.1371/journal.pone.0096228 2478865510.1371/journal.pone.0096228PMC4008525

[16] LeXF, MerchantO, BastRC, CalinGA, The Roles of MicroRNAs in the Cancer Invasion-Metastasis Cascade, Cancer Microenviron, 3 (2010) 137–147. doi: 10.1007/s12307-010-0037-4 2120978010.1007/s12307-010-0037-4PMC2990485

[17] SantarpiaL, NicolosoM, CalinGA, MicroRNAs: a complex regulatory network drives the acquisition of malignant cell phenotype, Endocr Relat Cancer, 17 (2010) F51–75. doi: 10.1677/ERC-09-0222 1984358010.1677/ERC-09-0222

[18] JiaZ, WangK, ZhangA, WangG, KangC, HanL, et al, miR-19a and miR-19b overexpression in gliomas, Pathol Oncol Res, 19 (2013) 847–853. doi: 10.1007/s12253-013-9653-x 2382491510.1007/s12253-013-9653-x

[19] VenturaA, YoungAG, WinslowMM, LintaultL, MeissnerA. ErkelandSJ et al,Targeted deletion reveals essential and overlapping functions of the miR-17~92 family of miRNA clusters, cell 132 (2008) 875–886. doi: 10.1016/j.cell.2008.02.019 1832937210.1016/j.cell.2008.02.019PMC2323338

[20] MuP, HanYC, BetelD, YaoE, SquatritoM, OgrodowskiP, et al, Genetic dissection of the miR-17~92 cluster of microRNAs in Myc-induced B-cell lymphomas, Genes Dev, 23 (2009) 2806–2811. doi: 10.1101/gad.1872909 2000893110.1101/gad.1872909PMC2800095

The article "MicroRNA-19a and microRNA-19b promote the malignancy of clear cell renal cell carcinoma through targeting the tumor suppressor RhoB" was retracted in 2026. Reasons: errors in the data; duplicated data; overlap with earlier publications; original data or images not available.

[21] CalinGA, LiuCG, SevignaniC, FerracinM, FelliN, DumitruCD, et al, MicroRNA profiling reveals distinct signatures in B cell chronic lymphocytic leukemias, Proc Natl Acad Sci U S A, 101 (2004) 11755–11760. doi: 10.1073/pnas.0404432101 1528444310.1073/pnas.0404432101PMC511048

[22] EadesG, YangM, YaoY, ZhangY, ZhouQ, miR-200a regulates Nrf2 activation by targeting Keap1 mRNA in breast cancer cells, J Biol Chem, 286 (2011) 40725–40733. doi: 10.1074/jbc.M111.275495 2192617110.1074/jbc.M111.275495PMC3220489

[23] XuXM, WangXB, ChenMM, LiuT, LiYX, JiaWH et al, MicroRNA-19a and -19b regulate cervical carcinoma cell proliferation and invasion by targeting CUL5, Cancer Lett, 322 (2012) 148–158. doi: 10.1016/j.canlet.2012.02.038 2256155710.1016/j.canlet.2012.02.038

[24] MendellJT, miRiad roles for the miR-17-92 cluster in development and disease, Cell, 133 (2008) 217–222. doi: 10.1016/j.cell.2008.04.001 1842319410.1016/j.cell.2008.04.001PMC2732113

[25] https://cancerstaging.org/references-tools/deskreferences/Pages/AJCC-7th-Ed-Cancer-Staging-Manual.aspx.

[26] RoosWP, KainaB, DNA damage-induced cell death: from specific DNA lesions to the DNA damage response and apoptosis, Cancer Lett, 332 (2013) 237–248. doi: 10.1016/j.canlet.2012.01.007 2226132910.1016/j.canlet.2012.01.007

[27] SahaiE, MarshallCJ, RHO-GTPases and cancer, Nat Rev Cancer, 2 (2002) 133–142. doi: 10.1038/nrc725 1263517610.1038/nrc725

[28] HuangM, PrendergastGC, RHOB in cancer suppression, histology and histopathology, 21(2006)213–218. doi: 10.14670/HH-21.213 1632904610.14670/HH-21.213

[29] ZhouJ, ZhuY, ZhangG, LiuN, SunL, LiuM, et al, A distinct role of RhoB in gastric cancer suppression, Int J Cancer, 128 (2011) 1057–1068. doi: 10.1002/ijc.25445 2047393310.1002/ijc.25445

[30] ZengPY, RaneN, DuW, ChintapalliJ, PrendergastGC, Role for RhoB and PRK in the suppression of epithelial cell transformation by farnesyltransferase inhibitors, Oncogene, 22 (2003) 1124–1134. doi: 10.1038/sj.onc.1206181 1260694010.1038/sj.onc.1206181

[31] QinS, AiF, JiWF, RaoW, ZhangHC, YaoWJ, miR-19a Promotes Cell Growth and Tumorigenesis through Targeting SOCS1 in Gastric Cancer, Asian Pacific Journal of Cancer Prevention, 14 (2013) 835–840. 2362124810.7314/apjcp.2013.14.2.835

[32] OtaA, TagawaH, KarnanS, TsuzukiS, KarpasA, KiraS, et al, Identification and Characterization of a Novel Gene, C13orf25, as a Target for 13q31-q32 Amplification in Malignant Lymphoma, cancer research,9(2004)3087–3095.10.1158/0008-5472.can-03-377315126345

